# Endothelial progenitor cell-derived exosomes, loaded with miR-126, promoted deep vein thrombosis resolution and recanalization

**DOI:** 10.1186/s13287-018-0952-8

**Published:** 2018-08-23

**Authors:** Jiacheng Sun, Zhiwei Zhang, Teng Ma, Ziying Yang, Jinlong Zhang, Xuan Liu, Da Lu, Zhenya Shen, Junjie Yang, Qingyou Meng

**Affiliations:** 1 Department of Vascular Surgery, The Second Affiliated Hospital of Soochow University, Suzhou, 215000 China; 2 Department of Biomedical Engineering, University of Alabama at Birmingham, Birmingham, 35294 Alabama USA; 3 Department of Cardiothoracic Surgery, The Second Affiliated Hospital of Soochow University, Suzhou, 215004 China; 4 Department of Cardiovascular Surgery of the First Affiliated Hospital and Institute for Cardiovascular Science, Soochow University, Suzhou, 215000 China

**Keywords:** Deep vein thrombosis, Resolution, Endothelial progenitor cell, Exosome, miR-126

## Abstract

**Background:**

Deep vein thrombosis (DVT) is caused by blood clotting in the deep veins. Thrombosis resolution and recanalization can be accelerated by endothelial progenitor cells. In this report, we investigated the effects of miR-126-loaded EPC-derived exosomes (miR-126-Exo) on EPCs function and venous thrombus resolution.

**Methods:**

In vitro promotional effect of miR-126-Exo on the migration and tube incorporation ability of EPCs was investigated via transwell assay and tube formation assay. In addition, a mouse venous thrombosis model was constructed and treated with miR-126-Exo to clarify the therapeutic effect of miR-126-Exo by histological analysis. Lastly, this study predicted a target gene of miR-126 using target prediction algorithms and confirmed it by luciferase activity assay, RT-qPCR, and Western blot.

**Results:**

Transwell assay and tube formation assay indicated that miR-126-Exo could enhance the migration and tube incorporation ability of EPCs. Moreover, in vivo study manifested enhanced thrombus organization and recanalization after miR-126-Exo treatment. Meanwhile, we identified that Protocadherin 7 as a target gene of miR-126.

**Conclusions:**

To sum up, our results demonstrated that EPC-derived exosomes loaded with miR-126 significantly promoted thrombus resolution in an animal model of venous thrombosis, indicating exosomes as a promising potential vehicle carrying therapeutic molecules for DVT therapy.

## Background

Deep vein thrombosis (DVT) is a complex event, accompanied by endothelial injury and blood flow turbulence. When the venous thrombi form, neutrophils and macrophages accumulate in the thrombi and extracellular matrices remodel. The resolution of venous thrombi requires the concordant action of different cell types [1]. In the initial stages of resolution, inflammatory cells infiltrate into the thrombus, clefts inside the thrombus enlarge and are lined by cells, and then new vessels generate through and around them. Therefore, neovascularization inside the thrombus is a critical event for thrombus resolution [2].

Evidences demonstrate that bone marrow-derived endothelial progenitor cells (EPCs) could largely contribute to thrombus resolution [3–5]. EPCs, first discovered by Asahara et al., could recruit to ischemic sites and help the neovascularization in ischemic areas [6]. Thousands of researches have proved the promotional effect of EPCs on angiogenesis in myocardial infarction, wound healing, and hind limb ischemia [7–9]. Our group and other researchers also reported the critical role of EPCs in thrombus resolution repeatedly. Modarai et al. first demonstrated the therapeutic effects of EPCs to resolve thrombi [3], and further confirmed by our group was that EPCs could recruit into resolving venous thrombi [10]. Our group utilized genetically modified EPCs, by vascular endothelial growth factor (VEGF) [11, 12] and miR-150 [13], respectively, to improve the effects of EPCs on thrombus resolution. However, more and more researches pointed out that EPCs exert their therapeutic effects mainly through secreting paracrine factors and the more recently studied exosomes [14, 15].

Exosomes are nano-sized extracellular vesicles, with a diameter of 30–100 nm, to mediate intercellular communication and modulate the function of recipient cells though delivery of proteins, RNA, microRNAs, and other molecular constituents [16]. Exosomes have now been recognized as a vehicle for intercellular communication since they have many remarkable attributes, such as stability, biocompatibility, and low immunogenicity [17]. miR-126 has been reported to be involved in maintenance of vascular integrity and angiogenesis, by repressing negative regulators of the VEGF pathway [18]. Mutation of miR-126 in mice caused leaky vessels, hemorrhaging, and partial embryonic lethality [18]. Our group demonstrated that upregulation of miR-126 contributes to endothelial progenitor cell function in deep vein thrombosis [19].

Given the transporting role of exosomes and the angiogenic potential of miR-126, in the present study we aimed to explore the effectiveness of miR-126-loaded exosomes derived from EPCs on thrombus resolution in an animal model of venous thrombosis.

## Methods

### Animals

C57/BL6 male mice were purchased from the Experiment Animal Center of Soochow University (Suzhou, China). All the procedures were approved by the Institutional Animal Care and Use Committee of Soochow University. The animals were maintained under a conventional state (12-h light/dark cycle) and fed with standard laboratory food and water.

### Culture and characterization of EPCs

EPCs were isolated from 4- to 6-week-old male mice as previously described [9]. Briefly, bone marrow-mononuclear cells (BM-MNCs) were collected from hipbones, femurs, tibiae, shoulder bones, ulnas, vertebra, and sternum, were separated and then smashed. BM-MNCs were further layered by density gradient centrifugation (Histopaque 1083, Sigma-Aldrich, St. Louis, MO, USA). After being washed twice, cells were cultured in Endothelial Cell Basal Medium-2 (EBM-2; Lonza, Basel, Switzerland), supplemented with EGM-2 MV Single Quots (Lonza, Basel, Switzerland) including VEGF, fibroblast growth factor-2 (FGF-2), epidermal growth factor (EGF), insulin-like growth factor (IGF), ascorbic acid, hydrocortisone, gentamycin, amphotericin-B, and 10% fetal bovine serum (FBS). Then, cells were incubated at 37 °C in a humidified atmosphere containing 5% CO_2_. The first medium change was performed to remove the nonadherent cells at 48 h, while adherent cells were further incubated in fresh EBM-2 MV. When grown to 90% confluence, cells were harvested with 0.25% trypsin (Sigma-Aldrich, St. Louis, MO, USA) and passaged continuously.

After the adherent mononuclear cells were washed twice by phosphate-buffered saline (PBS), 5 μg/ml of DiI-Ac-LDL solution (Biomedical Technologies Inc., Stoughton, MA, USA) was added into the medium and cultured away from light at 37 °C for 4 h. Then, the cells were fixed with 4% paraformaldehyde (PFA), and stained with 1 mg/mL DAPI (Invitrogen, Waltham, MA, USA) at room temperature for 15 min. The cells endocytosis of DiI-Ac-LDL was observed with a fluorescent microscope (Olympus, Tokyo, Japan). Further, the cells were identified by flow cytometry analysis. They were incubated with antibody against CD34, CD31, VE-cadherin, Flk-1, CD11b (FITC-conjugated anti-mouse), and CD45 (PE-conjugated anti-mouse) (BioLegend, San Diego, CA, USA). After being washed by 3% FBS/PBS, the expression of the surface markers of the cells were detected by quantitative fluorescence-activated cell sorting (FACS) using guava easyCyte 8 system (EMD Millipore, Burlington, MA, USA).

### Senescence-associated β-galactosidase assay

EPC senescence was determined by the number of senescence-associated β-galactosidase (SA-β-gal)-positive cells. SA-β-gal was stained using the senescence β-galactosidase staining kit (Beyotime Biotechnology, Shanghai, China), according to the manufacturer’s instructions. EPCs in passage 1 and passage 3 were used for this assay. The number of SA-β-gal-positive cells was determined by counting blue cells from at least 500 cells per field.

### Isolation, purification and characterization of EPC-derived exosomes

The EPCs were cultured in EBM-2 supplemented with EGM-2 MV Single Quots and 10% FBS, and the pre-existing exosomes in FBS were removed by ultracentrifugation at 110,000 g for 10 h. After 48 h, the culture supernatant was collected, and exosomes derived from EPCs (EPCs-exo) were separated from the medium using Total Exosome Isolation Reagent (Invitrogen, Waltham, MA, USA). According to the manual, the culture supernatant was centrifuged at 3000 g for 15 min to eliminate cells and debris. After that, Total Exosome Isolation Reagent was added to the supernatant with the ratio of 1:2. After being mixed well, the mixture was refrigerated at 4 °C overnight. Then, the steps below sequentially were: centrifugation of the mixture at 1500 g for 30 min, removal of the supernatant, again centrifugation of the residual solution at 1500 g for 5 min, and resuspension of the exosomes pellet with the appropriate buffer. Finally, EPCs-exo was stored at 80 °C for later use. The amount of EPC-derived exosome was detected by measuring the total protein content using a BCA protein assay kit (Beyotime Biotechnology, Shanghai, China).

Furthermore, EPC-derived exosomes were characterized by Western blot assay, transmission electron microscopy (TEM), and nanoparticle tracking analysis (NTA). Western blot assay was conducted as previously described using antibodies against CD63 and CD9 (Abcam, Cambridge, MA, USA), specific markers for exosomes were determined [20]. TEM was conducted by first resuspending purified exosomes in PBS and fixing it with 3% glutaraldehyde solution for half an hour at room temperature, then adding 20 ml of exosome to a copper grid and dying with 1% phosphotungstanic acid for 5 min at room temperature, and finally examining the dried grid using a Zeiss Libra 120 (Zeiss, Oberkochen, Germany) electron microscope at 120 kV. NTA was performed using a ZetaView PMX 120 (Particle Metrix, Dusseldorf, Germany) and its corresponding software (ZetaView) to automatically track and size purified exosomes simultaneously in real time according to the manufacturer’s instruction.

### Electroporation of microRNA-126 into exosomes

miR-126 mimics and miR-126 inhibitor and negative control RNA-oligonucleotides were purchased from Guangzhou Ribobio, Guangzhou, China. Electroporation of RNA-oligonucleotides into EPC-derived exosomes was performed using 4D-Nucleofector System Manual (Lonza, Basil, Switzerland) according to the manufacture’s instruction. Briefly, 10 μg exosome was precipitated and resuspended in 90 μl electroporation buffer of Lonza Cell Line Nucleofector Kit (Lonza, Basel, Switzerland), then mixed with 10 μl miR-126 mimics, miR-126 inhibitor or negative control before the mixture was transferred into cold 0.2 cm electroporation cuvettes and electroporated at 150 V/100 μF. After remove the free-floating miRNA, exosomes were re-isolated using ultracentrifugation. The final pellet (exosome) was resuspended in PBS, and stored at − 80 °C. RT-qPCR was performed to investigate the expression level of miR-126 in exosomes.

### Target gene prediction

Three target prediction algorithms—TargetScan (http://www.targetscan.org/), mirWALK (http://zmf.umm.uni-heidelberg.de/apps/zmf/mirwalk2/), and mircroRNA.org (http://www.mirtoolsgallery.org/miRToolsGallery/node/1055)—were used to predict the potential target relationship between miR-126 and protocadherin 7 (Pcdh7).

### Dual luciferase reporter assay

To elucidate whether Pcdh7 is a target gene of miR-126, wild-type (WT) and mutant seed regions of miR-126 in the 3′-UTR of Pcdh7 gene were cloned into pMIR-REPORT luciferase reporter plasmids (Invitrogen, Waltham, MA, USA). Plasmids with WT or mutant 3′-UTR DNA sequences were co-transfected with miR-126 mimics (100 nM; Sangon Biotech Co., Ltd., Shanghai, China) or negative control mimics into HEK293T cells (ATCC, Manassas, VA, USA). After cultivation at 37 °C for 24 h, cells were assayed using the dual luciferase assay system (Promega, Madison, WI, USA) according to the manufacturer’s instructions. All assays were repeated at least three times.

### In vitro transwell assay

The migratory ability of EPCs preconditioned with exosomes and/or recombinant Pcdh7 protein (Abcam, Cambridge, MA, USA) was assessed by the transwell assay, which was performed by using a chamber with 8 μm pore filter. In briefly, the EPCs were pretreated with 100 *μ*g Exo, miR-126-Exo or 25 *μ*l PBS for 24 h. In addition, the involvement of Pcdh7 for the role of miR-126 was also investigated. We compared the migratory ability of two groups of miR-126-Exo preconditioned EPCs treated with or without recombinant Pcdh7 protein. 1 μg of Pcdh7 protein was added to about 5 × 10^5^ cells EPCs pre-treated with 100 *μ*g miR-126-Exo. Then, cells (1 × 10^5^ cells), which were resuspended in 200 휇μl serum-free medium, were added into the upper chamber, and the lower chamber was filled with 0.5 ml culture medium including 10% FBS. Then, the chamber continued to incubate for 6 h routinely. And the non-migrating cells on the top side of the membrane were erased with cotton swabs. The migrating cells on the bottom of the membrane were fixed with 4% PFA, and then fluorescently stained with DAPI for 15 min at room temperature. After that, the cells were washed twice with PBS. The migratory staining cells were observed and counted by using a fluorescent microscope (Olympus, Tokyo, Japan).

### Tube formation assay (EPC incorporation assay)

The tube incorporation ability of EPCs preconditioned with exosomes was assessed by using human umbilical vein endothelial cells (HUVECs) and Matrigel as described previously [21]. In addition, the involvement of Pcdh7 for the role of miR-126 was also investigated using tube formation assay. Treatment of EPCs was described in the previous method. First, 1 μg/ml DiI was added into the EPCs culture, and culture continued at 37 °C for 20 min so as to label EPCs. Second, DiI-labeled EPCs (1000 cells) were mixed with HUVECs (20,000 cells) in 100 μl EGM-2MV Single Quots and 10% FBS. Third, 100 μl cell mixture was added into 50 μl Matrigel-(BioLegend, San Diego, CA, USA) coated wells in a 96-well plate, and continued to incubate for 6 h. Last, fluorescent microscope (Olympus, Tokyo, Japan) was applied to visualize and count the incorporated DiI-labeled EPCs, in order to evaluate the contribution of EPCs to EC-derived tube formation.

### Mouse model of deep venous thrombosis and exosome therapy

The model of laminated thrombus was established in the inferior vena cava of the C57/BL6 male mice using FeCl_3_ as described previously with a little modification [19]. In brief, after anesthesia, a mid-abdominal incision was performed, and the inferior vena cava between the renal vein and the iliac vein was carefully exposed by wet cotton swabs. The inferior vena cava was encircled by a narrow strip of wet filter paper for 30 s, which was pre-soaked by 15% FeCl_3_ solution. 300 *μ*g of Exo or miR-126-Exo were transplanted into the femoral vein in situ. The experimental mice were divided into three groups: NC group (control, *n* = 5), Exo group 2 (treated with empty exosome, n = 5), and miR-126-Exo group (treated with exosome transfected with miR-126 mimics, n = 5).

Animals were sacrificed at 14 days post-operation. The thrombus together with surrounding venous wall was harvested. The specimens along the whole thrombus were fixed with 4% paraformaldehyde, embedded in paraffin, sliced 5 μm sections, and conducted with hematoxylin and eosin (HE) staining and immunofluorescent staining.

### Histological examination

Animals were sacrificed at 14 days post-operation. The thrombus together with surrounding venous wall was harvested. The specimens along the whole thrombus were fixed with 4% paraformaldehyde, embedded in paraffin, sliced 5 μm sections, and conducted with HE staining and immunofluorescent staining. Immunofluorescent staining against CD31, a sort of endothelial cells specific surface marker, was performed to illustrate the neovascularization in venous thrombus. The images of sections were taken by light microscopy (Nikon, Tokyo, Japan). The size of thrombus was quantified by measuring the area of each thrombus section using the image-analysis software (Image-Pro Plus, Media Cybernetics, Rockville, MD, UK). The newborn capillaries accounted for vascular recanalization were detected by counting the number of the CD31^+^ cells in 5 random fields under the light microscopy (Nikon, Tokyo, Japan).

### Quantitative real-time PCR assay

To further determine the potential target relationship between miR-126 and Pcdh7, EPCs were treated with 100 μg Exo transfected with miR-126 mimics or miR-126 inhibitor, or PBS for 48 h. In addition, the mRNA expression level of miR-126 and Pcdh7 in thrombosis mouse model after miR-126-Exo treatment for 14 days was detected. Total RNA was extracted from the sample using the PureLink RNA Mini Kit (Ambion, Life Technologies, Waltham, MA, USA), according to the manufacturer’s specifications. Briefly, total RNA was reverse translated to cDNA using the PrimeScript RT reagent Kit (Takara, Tokyo, Japan). Through quantitative real-time PCR (qRT-PCR) using SYBER Green (Applied Biosystems, Foster City, CA, USA) and the StepOne-Plus real-time PCR system (Applied Biosystems, Foster City, CA, USA), the cDNA was dramatically amplified with the gene-specific primers. GAPDH and U6 were used as normalization to the expression levels of Pcdh7 and miR-126, respectively. For exosomes, procedures of RT-qPCR were basically identical except U6 was used to normalize the results. The 2 − ΔΔCT method was used to evaluate the relative quantification of changes in the expression of target genes. Every primer of RT-qPCR was repeated in triplicate, and the mean values were presented as the gene expression levels. The primers used in RT-qPCR were listed in Table 1.

**Table 1:** Primer sequences for quantitative real-time PCR

Gene name	Forward primer (5′-3′)	Reverse primer (5′-3′)
GAPDH	TGTGTCCGTCGTGGATCTGA	ACCACCTTCTTGATGTCATCATACTT
Pcdh7	ATGCTGAGGATGCGGACCA	CTACAGATAAACTTCTCTTCTAGTG

### Western blot

The expression of bovine serum albumin (BSA) in exosomes samples were determined using Western blot to identify whether exosomes from FBS were totally eliminated. In addition, EPCs treated with Exo transfected with miR-126 mimics or miR-126 inhibitor, or PBS were also used to determine the expression level of Pcdh7 protein. The protein was extracted from exosomes, FBS and cells, which were lysed with M-PER reagents and Halt Protease Inhibitor Cocktail kits (Pierce Biotechnology, Waltham, MA, USA). The concentration of extracted protein was detected by BCA Protein Assay Kit (Beyotime Biotechnology, Haimen, China). Then, the extracted protein was separated by 10% SDS-PAGE and transferred to nitrocellulose membrane (EMD Millipore, Burlington, MA, USA). The membranes were blocked using Tween 20/PBS including 5% skim milk, and then incubated with primary antibody against Pcdh7 (1:100, Abcam, Cambridge, MA, USA) and β-actin (1:1000, Beyotime Biotechnology, Haimen, China) and followed by the HRP-conjugated secondary antibody (1:1000; Beyotime Biotechnology, Haimen, China). The protein-labeled bands were determined using the enhanced chemiluminescent kit and analyzed using the Scion Image Software (Scion, Torrance, CA, USA). The intensity of protein bands was evaluated with Image J (National Institutes of Health, Bethesda, MD, USA). The intensity of the protein bands was quantified relative to the β-actin bands from the same sample.

### Statistical analysis

All data are expressed as mean ± standard deviation (SD). Comparisons between two groups were assessed by the Mann-Whitney *U* test, and one-way ANOVA was used to compare among groups. *P* < 0.05 was considered as statistical significance. Statistical analysis was taken place using the statistical software GraphPad Prism 6.0. (GraphPad Software, San Diego, CA, USA),

## Results

### Characterization of EPCs

EPCs were isolated from bone marrow of C57BL/6 mice as described previously. Adherent cells changed their morphology into typical spindle-shape at day 3 and formed colonies at day 7 (Fig. 1a). DiI-Ac-LDL uptake assay was further conducted to determine the characterization of EPCs, showing that EPCs could specifically uptake DiI-Ac-LDL as previously reported (Fig. 1b) [9]. Moreover, flow cytometry was used to identify the surface antigens of EPCs. Results showed that EPCs were positive for CD34, CD31 and VE-Cadherin, while negative for Flk-1, CD11b and CD45 (Fig. 1c).

**Fig. 1:** Characterization of EPCs and senescence detection of EPCs. **a** Spindle-shaped EPCs were observed at day 3 and formed colonies at day 7 after plating BM-MNCs. Bar, 50 μm. **b** EPCs uptaken DiI-Ac-LDL could be visualized (*red*). DAPI was used to stain the nucleus (*blue*). Bar, 25 μm. **c** Phenotypic analysis of cell surface markers of EPCs by flow cytometry. **d** Senescent cells were labeled as *blue* using senescence β-galactosidase staining kit. **e** Quantitative analysis of senescent EPCs in passage 0 and passage 2 (*n* = 3)

### No difference between senescence of passage 1 and passage 3 EPCs

Considering senescence phenomena induced by in vitro cultivation could alter the cell functions as well as paracrine effect [22], we performed senescence-associated beta-galactosidase assay to determine the senescence of EPCs in different passages. As shown in Fig. 1d, the senescent EPCs could be visualized in blue color. The statistical analysis (Fig. 1e) shown the senescent ratio in passage 1 EPCs and passage 3 EPCs revealed no significant differences between different passages (passage 1 EPCs: 7.467% ± 0.7623% vs. passage 3 EPCs: 7.667% ± 1.342%; *n* = 3; *P* = 0.90).

### Characterization of EPC-derived exosomes

Exosomes derived from EPCs were also determined using to biochemical and biophysical analyses. Western blotting result identified that EPC-derived exosomes were negative of expressing bovine serum albumin, which indicated that exosomes in FBS were completely eliminated by ultracentrifugation (Fig. 2a). In addition, Western blot result showed that EPC-derived exosomes were positive for CD9 and CD63 (Fig. 2b). Electron microscopy analysis of exosomes exhibited typical cup-shaped morphology (Fig. 2c). The exosomes were morphology homogenous with ranging in size from 80 to 150 nm and peaking at 98 nm as examined by nanoparticle tracking analysis (Fig. 2d). Furthermore, RT-qPCR result suggested that miR-126 expression in EPC-derived exosomes was significant elevated after electroporated with miR-126 mimics and dramatically decreased when transferred with miR-126 inhibitor, respectively (*P* < 0.05; Fig. 2e).

**Fig. 2:** Characterization of EPC-derived exosomes. **a** Western blot analysis of bovine serum albumin (BSA) expression in fetal bovine serum (FBS) and EPC-derived exosomes. **b** Western blot analysis of EPC-derived exosomes by CD63 and CD9. **c** Transmission electron microscope (TEM) images of EPC-derived exosomes. Bar, 250 nm. **d** Size distribution of EPC-derived exosomes measured by nanoparticle tracking analysis (NTA) peaking at 98 nm. **e** RT-qPCR result identified the up- and downregulation of miR-126 in exosomes transfected with miR-126 mimics or inhibitor, respectively (n = 3). ***P < 0.001

### Pcdh7 is a target gene of miR-126

Three databases (TargetScan, microRNA, and miRDB) were used to predict the target gene of miR-126, among those we chose Protocadherin 7 (Pcdh7) as the candidate target gene. miR-126 was predicted capable of binding on the 3’-UTR of Pcdh7 as shown in Fig. 3a. We constructed the luciferase reporter vector (Fig. 3b) to perform the luciferase reporter assay. As shown in Fig. 3c, miR-126 significantly reduced the relative luciferase reporter activity of the wild-type Pcdh7 3′ -UTR, whereas that of the mutant Pcdh7 3′ -UTR did not change obviously, which suggests that miR-126 could directly bind to the 3′ -UTR of Pcdh7.

**Fig. 3:** Pcdh7 is a putative target of miR-126 in EPCs. **a** Binding motif (8471–8474, 8480–8485) of miR-126 on Pcdf7 3′-UTR (4793–8695). **b** Construction of luciferase construct. **c** Relative Rluc/Luc ratio (n = 3). **d** mRNA expression of Pcdh7 in EPCs after transfection of miR-126 mimics and inhibitors (*n* = 6). **e** Pcdh7 protein expression level in EPCs after transfection of miR-126 mimics and inhibitors. **f** Qualification of protein expression level (*n* = 4). **P < 0.01, ***P < 0.001

We further confirmed this hypothesis by determining the Pcdh7 expression level in EPCs transfected with miR-126 mimics or miR-126 inhibitor. RT-qPCR result revealed that Pcdh7 expression level has decreased by 69.70% after overexpression of miR-126 (*P* < 0.01) while presenting higher expression level in the miR-126 inhibitor group compared with the control group (Fig. 3d). Western blot results indicated that Pcdh7 protein level also presented similar changes as Pcdh7 mRNA, presenting a negative correlation with the expression level of miR-126 (Fig. 3e, f). These results provided clear evidence that Pcdh7 is a putative target of miR-126.

### In vitro migration ability of EPCs was elevated by exosomes transfected with miR-126

The function of miR-126-Exo or Exo on the migration ability of EPCs was detected by a transwell system. EPCs were co-culture with miR-126-Exo or Exo for 24 h before seeded on the upper chamber, respectively. Cells were stained by DAPI and observed in HPFs (Fig. 4a). After treatment with miR-126-Exo or Exo, EPCs both manifested augmented migration ability compared with control group, respectively (Fig. 4b; miR-126-Exo group 122.00 ± 23.43/HPF vs. NC group 36.33 ± 4.04/HPF, *P* < 0.05; Exo group 78.33 ± 3.22/HPF vs. NC group 36.33 ± 4.04/HPF, *P* < 0.05). Furthermore, miR-126-Exo group exhibited even more migrated cells than Exo group (*P* < 0.001). This assay indicated that EPC-derived exosomes exert promotional effect on migration ability of EPCs, and miR-126 overexpressed exosome could expand this promotional effect.

**Fig. 4:** Migration and tube incorporation ability of EPCs was elevated by miR-126-loaded exosomes. **a** Representative images show DAPI-stained EPCs (*blue*). Bar, 100 μm. **b** Number of migrated cells was calculated manually and presented as mean ± SD (n = 4). **c** DiI-positive incorporated EPCs could be observed in the HUVEC-formed tube structure. Bar, 200 μm. **d** Number of DiI-positive incorporated EPCs was counted and presented as mean ± SD (n = 4). *P < 0.05, **P < 0.01, ***P < 0.001

### Incorporation ability of EPCs into tube structure was promoted by miR-126-Exo

Angiogenesis potential of EPCs was studied by tube formation assay according to former reports. EPCs could integrate into the tube-like structure formed by HUVECs but forming vessels independently. As shown in Fig. 4c, DiI-labeled EPCs (red color) in Exo group were significantly ascended than NC group, whereas incorporated EPCs in miR-126-Exo group were more than Exo group. Precisely, as shown in Fig. 4d, 23.42 ± 1.33/HPF and 35.01 ± 9.96/HPF incorporated EPCs were counted in Exo and miR-126-Exo groups, respectively, whereas only 16.75 ± 0.83/HPF cells were observed in NC group.

### Involvement of Pcdh7 for the role of miR-126

We further determined that whether the elevation of migration ability and tube incorporation ability of EPCs treated with miR-126-Exo could be counteracted by Pcdh7. We treated miR-126-Exo preconditioned EPCs with recombinant Pcdh7 protein, then performed transwell assay and tube formation assay. As shown in Fig. 5, the migrated EPCs and incorporated EPCs were obviously decreased after Pcdh7 treatment. Specifically, migrated EPCs drop from 65.98 ± 2.534 cells per HPF to 18.96 ± 4.985 cells per HPF (*N* = 3; *P* < 0.01; Fig. 5b) after co-culture with recombinant Pcdh7 protein; incorporated EPCs decreased from 42.50 ± 4.406 cells/mm tube length to 24.25 ± 2.394 cells/mm tube length (*N* = 3; *P* < 0.05; Fig. 5d). These results indicated that the existence of Pcdh7 could counterbalance the effect of miR-126-Exo.

**Fig. 5:** investigation of the involvement of Pcdh7 on the role of miR-126 using transwell assay and tube formation assay. **a** Representative images show migrated EPCs (*blue*) were decreased by the application of recombinant Pcdh7 protein. Bar, 100 μm. **b** Number of migrated cells was calculated manually and presented as mean ± SD (n = 3). **c** Decreased DiI-positive incorporated EPCs were observed in the HUVEC-formed tube structure after Pcdh7 treatment. Bar, 200 μm. **d** Number of DiI-positive incorporated EPCs was counted and presented as mean ± SD (n = 3). *P < 0.05, **P < 0.01

### miR-126 loaded exosomes augmented thrombus organization and recanalization

It has been proven that thrombus organization and recanalization is involved in the dynamic and complex pathophysiologic process of deep vein thrombosis [23]. We then performed HE staining and immunofluorescent staining to examine the effect of miR-126-Exo on thrombus organization and recanalization in mouse model, respectively.

Fourteen days after the treatment of miR-126-Exo or Exo, inferior vena cave was removed and HE staining was conducted (Fig. 6a). Typical thrombus organization could be observed within vessel cavity in NC and Exo groups where red blood cells, platelets and fibrin stained dried red with dried blue-colored nucleated cells, including ECs, monocytes, and neutrophil granulocytes entered into the center of thrombus. In contrast, more nucleated cells and obvious channels were observed in miR-126-Exo group, presenting downscaled thrombi size and a large number of newborn vessels.

**Fig. 6:** Histological analysis of thrombus in mouse DVT model. **a** Representative images of HE staining for the thrombus sections. *Arrows* indicated the recanalization in thrombus. Bar, 200 μm. **b** Representative images of CD31 staining for the thrombus sections. *Arrows* indicate the new-formed vessels with CD31 expression. Bar, 50 μm. **c** CD31-positive vessels were manually counted and presented as mean ± SD (n = 3). **d**, **e** Expression level of miR-126 and Pcdh7 mRNA in thrombus 14 days post-operation. *P < 0.05, **P < 0.01, ***P < 0.001

A common cell-surface marker for capillary ECs, CD31, was detected to validate the recanalization of the thrombus. DAPI was used for the indication of cell nuclei. As the arrows marked in Fig. 6b, a green-florescent ring structure could be identified as newborn capillaries located at the perimeter of thrombus, which is consistent with HE staining. By day 14, a larger number of newborn vessels were identified in miR-126-Exo group in comparison with Exo group and NC group (Fig. 6c; miR-126-Exo group 29.83 ± 9.96/HPF vs. Exo group 23.42 ± 1.33/HPF, *P* < 0.001; miR-126-Exo group 29.83 ± 9.96/HPF vs. NC group 4.50 ± 1.05/HPF, *P* < 0.001). These results indicated that miR-126 overexpressed exosomes exerted curative effects by ameliorating thrombus organization and recanalization.

### Pcdh7 mRNA expression was elevated in thrombus treated with miR-126-Exo

In vitro study has revealed miR-126 could enhance the migration and angiogenic effect of EPCs by targeting to Pcdh7. We further studied whether miR-126 exerted the curative effect on thrombus by targeting to Pcdh7 in vivo. Thrombus in inferior vena cava were harvested 14 days post-operation. RT-qPCR was conducted to determine the expression level of miR-126 and Pcdh7 mRNA. As shown in Fig. 6d, miR-126 expression level was dramatically elevated in the miR-126-Exo-treated group compared with both the NC group and Exo group (both *P* < 0.05; NC group: 1.04 ± 0.04; Exo group: 1.58 ± 0.33; miR-126-Exo group: 5.39 ± 1.94; *n* = 3). Consistently, Pcdh7 mRNA expression in the miR-126-Exo group was increased by approximately 1.5-fold compared with NC group (Fig. 6d; *P* < 0.01; *n* = 3).

## Discussion

In this study, we demonstrated that EPC-derived exosomes loaded with miR-126 significantly promoted thrombus resolution in an animal model of venous thrombosis. In vitro, miR-126-exosomes enhanced migration and angiogenesis in EPCs. These findings greatly extend our current understanding of exosomes on neovascularization, indicating exosomes as promising vehicles of therapeutic molecules for the treatment of thrombus.

Deep vein thrombosis (DVT) occurs when the blood clotted in the deep veins, usually in the legs, which eventually causes leg pain or swelling and even pulmonary embolism. Pulmonary embolism often leads to sudden unexpected death. Thrombus resolution is a tissue repair process involving inflammation, proliferation, and maturation phases. Recently, accumulating evidence demonstrated that bone marrow-derived stem/progenitor cells play crucial roles in tissue repair, such as skin wound healing, myocardial infarction and thrombus resolution [4, 24, 25]. Dr. Alberto Smith reported that thrombus failed to resolve in urokinase-type plasminogen activator knockout mice but was rescued by transplantation of normal bone marrow cells [26], which gave solid evidence for the thrombus-resolving role of the cells. Dr. Asahara demonstrated that endothelial progenitor cells were found in the thrombus at 7 days, and differentiated into mature endothelium forming the vascular channels inside the thrombi [27]. The clinical study performed by Dr. Han proved that EPCs promoted the recanalization of thrombi in the damaged vessels for patients with DVT [28].

In our previously reports, we overexpressed miR-126 in EPCs and demonstrated that miR-126 could enhance EPCs’ migration and tubulogenic activity in vitro, and could promote EPCs’ homing and thrombus resolving in vivo [19]. In addition, more and more researches pointed out that EPCs exert the therapeutic effects mainly through secreting paracrine factors and exosomes, which is a research hotspot recently. We propose that EPC-derived exosomes, loaded with therapeutic miR-126, could play a crucial role in the resolution of thrombus. In the present study, we demonstrated that miR-126-mimics-exosomes could promote the migration and angiogenesis of EPCs. Most importantly, miR-126-exosomes significantly improved thrombus organization and recanalization in mouse DVT models. Further, we investigated the potential mRNA targets of miR-126 by online database. Protocadherin 7 (Pcdh7) is a target of miR-126 predicted by bioinformatics. We confirmed this relationship using luciferase reporter assay, qPCR and Western blot. We demonstrated that the existence of recombinant Pcdh7 protein could counterbalance the effect of miR-126-Exo on the migration and tube incorporation ability of EPCs in vitro. This result provided solid evidence that miR-126 exerts its effects by inhibiting Pcdh7 expression. In addition, we detected the miR-126 and Pcdh7 mRNA expression level in thrombus 14-day post-operation, miR-126 level presented a significant elevation in miR-126-Exo group whereas Pcdh7 mRNA level was decreased. The enhanced thrombus recanalization and organization in miR-126-Exo group could be attributed to the inhibition of Pcdh7 expression. Consistently, previous reports [29, 30] have indicated that Pcdh7 is reversely correlated with angiogenesis, which could explain that angiogenesis is promoted by miR-126 mimics.

## Conclusions

In conclusion, our results demonstrated that EPC-derived exosomes loaded with miR-126 significantly promoted thrombus organization and recanalization in an animal model of venous thrombosis. Thus, we may reasonably speculate that exosomes may be a promising potential vehicle carrying therapeutic molecules for DVT therapy.

## Abbreviations

BM-MNCs: Bone marrow-mononuclear cells
DVT: Deep vein thrombosis
EGF: Epidermal growth factor
EPC: Endothelial progenitor cells
Exo: Exosomes
FACS: Fluorescence-activated cell sorting
FBS: Fetal bovine serum
FGF-2: Fibroblast growth factor-2
HUVEC: Human umbilical vein endothelial cell
IGF: Insulin-like growth factor
NTA: Nanoparticle tracking analysis
PBS: Phosphate-buffered saline
Pcdh7: Protocadherin 7
SD: Standard deviation
TEM: Transmission electron microscopy
VEGF: Vascular endothelial growth factor
WT: Wild-type
